The article "Effects of Minocycline on Cognitive Impairment, Hippocampal Inflammatory Response, and Hippocampal Alzheimer's Related Proteins in Aged Rats after Propofol Anesthesia" was retracted in 2023. Reasons: suspected computer-generated content; unreliable results or conclusions; concerns about the data; concerns about the results or conclusions.

# Effects of Minocycline on Cognitive Impairment, Hippocampal Inflammatory Response, and Hippocampal Alzheimer's Related Proteins in Aged Rats after Propofol Anesthesia

**DOI:** 10.1155/2022/4709019

**Published:** 2022-04-26

**Authors:** Xuemei Liang, Rong Zhang

**Affiliations:** ^1^Department of Neurology, Tianjin Fourth Central Hospital, Tianjin 300140, China; ^2^Department of Neurology, Xianyang Hospital of Yan 'an University, Xianyang Shanxi 712000, China

## Abstract

The aim of this study was to evaluate the effect of minocycline preadministration on cognitive dysfunction, hippocampal inflammatory response, and hippocampal senile dementia-related proteins induced by propofol anesthesia in aged rats. Sixty male SD rats, aged 20 months and weighing 340-410 g, were randomly divided into three groups: normal saline (NC) group, propofol group (prop), and minocycline (M) group. Prop group rats were injected intraperitoneally with 100 mg/kg propofol. The rats in group M were injected intraperitoneally with 50 mg/kg minocycline 30 minutes before injection of 100 mg/kg propofol, and the rest were the same as prop group. The rats in NC group were received intraperitoneal injection of the same amount of normal saline. The results indicated that compared with group C, the expressions of GSK-3*β*, acetyl-NF-*κ*B (Lys310), Tau, and Amlyoid-beta were upregulated, the levels of TNF-*α*, IL-1*β*, and IL-6 were increased, the escape incubation period was prolonged, and the exploration time was shortened in prop group, while the expression of GSK-3*β*, acetyl-NF-*κ*B (Lys310), Tau, and Amlyoid-beta in minocycline group was downregulated, the levels of TNF-*α*, IL-1*β*, and IL-6 were decreased, the escape incubation period was shortened, and the exploration time was shortened. In conclusion, preadministration of minocycline can improve cognitive impairment induced by propofol anesthesia in aged rats, and its mechanism of action may be related to minocycline inhibiting hippocampal inflammatory reaction and downregulating the expression of GSK-3*β*, acetyl-NF-*κ*B (Lys310), Tau, and Amlyoid-beta proteins in hippocampus.

## 1. Introduction

Postoperative cognitive dysfunction (POCD) is a common complication after surgery. Its clinical symptoms mainly include hypomnesis, inattention, decreased language understanding, and decreased social communication ability. Its clinical symptoms often occur within a few days to weeks after surgery and can last for a long time [1, 2]. The pathogenesis of POCD is very complex and has not yet been clearly clarified. Anesthetics are considered to be the main cause of POCD [3]. Propofol is a commonly used intravenous anesthetic, which takes effect by activating aminobutyric acid receptor-chloride ion complex [4]. Propofol takes effect quickly, the induction period is short and stable, the awakening is fast, and the probability of complications such as nausea and vomiting after operation is low. Propofol is commonly used for induction and maintenance of anesthesia and sedation of critically ill patients [5]. However, some studies have shown that propofol can change the phosphorylation level of Tau protein in hippocampus and lead to the occurrence of POCD, but its pathogenesis is still unclear [6]. Studies have shown that central nervous inflammation plays an important role in POCD [7].

The article "Effects of Minocycline on Cognitive Impairment, Hippocampal Inflammatory Response, and Hippocampal Alzheimer's Related Proteins in Aged Rats after Propofol Anesthesia" was retracted in 2023. Reasons: suspected computer-generated content; unreliable results or conclusions; concerns about the data; concerns about the results or conclusions.

Cognitive function refers to the brain's ability to acquire, store, process, and extract information, that is, the ability to grasp the composition of things, the performance of things, the relationship between things and other things, the development power and direction of things, and the basic laws, mainly including learning, memory, language, execution, calculation, and judgment. Studies have shown that the brain region most closely related to cognitive functions such as spatial learning and memory is hippocampus [8, 9].

Minocycline is a new broad-spectrum tetracyclic antibiotic. Studies have found that it plays a brain protective role in various neurodegenerative diseases such as Alzheimer's disease and Parkinson's disease, showing that it has neuroprotective effects such as antiapoptosis and anti-inflammation [10, 11]. Minocycline can reach a high concentration in the nerve center and is one of the few antibiotics that can penetrate the blood-brain barrier. Therefore, it can play a central anti-inflammatory role, reduce the production of central inflammatory factors, and thus play a brain-protective role [12]. However, it is still unclear whether minocycline can improve the cognitive dysfunction induced by propofol anesthesia in rats, and whether its mechanism of action is related to horse inflammatory response and hippocampal senile dementia-related proteins.

Tau protein is a low molecular weight glycoprotein mainly distributed in central nervous cells. When Tau protein is highly phosphorylated and abnormally glycosylated, Tau protein loses its stabilizing effect on microtubules and damages the function of nerve fibers [13]. Some studies believe that hyperphosphorylation of Tau protein in hippocampus is related to cognitive dysfunction [14]. Some studies have shown that general anesthetic drugs can increase the expression of Tau and Amyloid-beta proteins in hippocampus, inducing or aggravating the occurrence of postoperative cognitive dysfunction [15].

Glycogen synthase and enzyme-3*β* (GSK-3*β*) participate in the regulation of hippocampal synaptic plasticity [16]. Some studies have shown that the activation of GSK-3*β* and acetyl-NF-*κ*B (Lys310) in hippocampus is related to the formation of memory [17, 18].

The article "Effects of Minocycline on Cognitive Impairment, Hippocampal Inflammatory Response, and Hippocampal Alzheimer's Related Proteins in Aged Rats after Propofol Anesthesia" was retracted in 2023. Reasons: suspected computer-generated content; unreliable results or conclusions; concerns about the data; concerns about the results or conclusions.

Therefore, this study observed the effect of minocycline on POCD induced by propofol anesthesia in rats. The possible mechanism of action was discussed from the mRNA expression and content of hippocampal glycogen synthetase and enzyme-3*β* (GSK-3*β*) and acetyl-NF-*κ*B (Lys310), hippocampal Tau protein, Amyloid-beta protein, hippocampal TNF-*α*, IL-1*β*, and IL-6, to provide new strategies and targets for prevention and treatment of POCD.

## 2. Materials and Methods

### 2.1. Animal Selection and Grouping

Sixty male specific pathogen free (SPF) SD rats, aged 20 months and weighing 340-410 g, were randomly divided into three groups (*n* = 20): normal saline (NC) group, propofol group (prop), and minocycline (M) group. Prop group rats were injected intraperitoneally with 100 mg/kg propofol. The rats in group M were injected intraperitoneally with 50 mg/kg minocycline 30 minutes before injection of 100 mg/kg propofol, and the rest were the same as prop group. NC group was given intraperitoneal injection of the same amount of normal saline. Arterial blood gas analysis was performed immediately after anesthesia. Hippocampal tissues were taken 24 hours after anesthesia. Western blot was used to determine the expressions of hippocampal glycogen synthetase and enzyme-3*β* (GSK-3*β*) and acetyl-NF-*κ*B (Lys310), hippocampal Tau protein, and Amyloid-beta protein. Real-time quantitative PCR and ELISA were used to detect the mRNA expression and content of hippocampal TNF-*α*, IL-1*β*, and IL-6, respectively. Cognitive function was evaluated on the 2nd day after anesthesia. The protocol of current study was approved by institutional ethical committee of our hospital.

### 2.2. Analysis of Blood Glucose and Arterial Blood Gas

Immediately after anesthesia, 5 rats in each group were randomly selected, 200 *μ*L of left ventricular blood was immediately taken with needle 32, blood sugar level was measured by ABL-800FLEX analyzer, and arterial blood gas analysis was carried out.

### 2.3. Determination of Hippocampal Associated Proteins

Hippocampal tissues of 5 rats were randomly selected 24 hours after anesthesia. Western blot was used to detect the expression of glycogen synthetase, GSK-3*β*, acetyl-NF-*κ*B (Lys310), Tau protein, and Amyloid-beta protein in hippocampus. Hippocampal tissue homogenate was taken and centrifuged, supernatant was taken, and protein was quantified by Bradford method and stored at -80°C for later use. Samples were electrophoresis on 10% sodium dodecyl sulfonate-polyacrylamide gel and then electronically transferred to PVDF membrane. After blocking with 5% skimmed milk, the primary antibodies against GSK-3*β* (CST, USA), acetyl-NF-*κ*B (Lys310, Abcam, USA), Tau (CST, USA), Amlyoid-beta (Abcam, USA), and HRP-labeled sheep anti-mouse (ProteinTech, China) or anti-rabbit secondary antibodies (Protein Tech, China) were added successively. DAB chromogenic agent (Transgene, China) was used for color development. Image Lab 3.0 software was used for gray analysis, and the ratio of the gray value of the target protein to the gray value of-actin was used to reflect the expression level of the protein.

The article "Effects of Minocycline on Cognitive Impairment, Hippocampal Inflammatory Response, and Hippocampal Alzheimer's Related Proteins in Aged Rats after Propofol Anesthesia" was retracted in 2023. Reasons: suspected computer-generated content; unreliable results or conclusions; concerns about the data; concerns about the results or conclusions.

### 2.4. mRNA Determination of TNF-*α*, IL-1*β*, and IL-6 in Hippocampus

The hippocampal tissues of 5 rats were randomly selected 24 hours after anesthesia. Total RNA was extracted from hippocampal tissues and reverse transcribed. Real-time fluorescence quantitative PCR was performed to detect the mRNA expression levels of TNF-*α*, IL-1*β*, and IL-6. The target gene-specific primer was designed and synthesized by Takara Company. TNF-*α* upstream primer: 5′-AACT-GGCAGAGGAGGCG-3′, downstream primer: 5′-CAGAAGAGCGTGGTGGC-3′; IL-1*β* upstream primer: 5′-GTGGGATGAT-GACGACC-3′, downstream primer: 5′-CAGAATTGCCATTG-CACAAC-3′; IL-6 upstream primer: 5′-CCGGAGAGGAGACT-TCACAG-3′, downstream primer: 5′-CAGAATTGCCATTG-CACAAC-3′; GAPDH upstream primer: 5′-CCCCCAATG-TATCCGTTGTG-3′, downstream primer: 5′-TAGCCCAGGATGC-CCTTTAGT-3′. The 2^-△△Ct^ method was used to calculate that relative expression level of the target gene mRNA.

### 2.5. Determination of TNF-*α*, IL-1*β*, and IL-6 in Hippocampus

Five rats in each group were randomly selected 24 hours after anesthesia, hippocampus tissue was separated, hippocampus tissue homogenate was centrifuged, and supernatant was taken. The contents of TNF-*α*, IL-1*β*, and IL-6 in hippocampus tissue were determined by ELISA.

### 2.6. Determination of Cognitive Function

Another 10 rats were taken and returned to the cage after fully awake. Morris water maze (MWM) test was carried out on the 2nd day after anesthesia. Ethovision animal movement track recording system automatically records the swimming track of rats. Taking the time from entering the water to climbing the platform as the escape incubation period, the daily test average was taken. Rats that could not find the platform within 60 seconds were placed on the platform, and the escape incubation period was recorded as 60 seconds. The rats were trained continuously for 5 days, and the escape incubation period was recorded. On the 7th day, the platform was removed. Rats were put into the water from the same water entry point facing the pool wall, and the exploration time (the residence time of rats in the quadrant where the platform is located within 60s) was recorded.

The article "Effects of Minocycline on Cognitive Impairment, Hippocampal Inflammatory Response, and Hippocampal Alzheimer's Related Proteins in Aged Rats after Propofol Anesthesia" was retracted in 2023. Reasons: suspected computer-generated content; unreliable results or conclusions; concerns about the data; concerns about the results or conclusions.

### 2.7. Statistical Treatment

SPSS 25.0 statistical software was used for analysis. The measurement data were expressed as mean ± standard deviation. The comparison among groups was conducted by single factor analysis of variance with LSD test. The one-sided *P* value less than 0.05 was statistically significant.

## 3. Results

### 3.1. Comparison of Arterial Blood Gas Index and Blood Glucose of Rats in Each Group

There was no significant difference in blood pH, PaCO_2_, PaO_2_, and blood glucose among NC group, prop group, and minocycline group (*P* > 0.05), as shown in Table 1.

### 3.2. Comparison of GSK-3*β* and Acetyl-NF-*κ*B (Lys310) Protein Expression in Hippocampus of Rats in Each Group

Compared with NC group, the expression of GSK-3*β* and acetyl-NF-*κ*B (Lys310) in hippocampus of prop group rats was upregulated (*P* < 0.05); compared with prop group, the expression of GSK-3*β* and acetyl-NF-*κ*B (Lys310) protein in hippocampus of minocycline group rats was downregulated (*P* < 0.05), as shown in Figure 1.

### 3.3. Comparison of Tau and Amlyoid-Beta Protein Expression in Hippocampus of Rats in Each Group

Compared with NC group, the expression of Tau and Amlyoid-beta protein in the hippocampus of prop group rats was upregulated (*P* < 0.05); compared with prop group, the expression of Tau and Amlyoid-beta protein in hippocampus of minocycline group rats was downregulated (*P* < 0.05), as shown in Figure 2.

### 3.4. Comparison of TNF-*α*, IL-1*β*, and IL-6 Contents and mRNA Expression in Hippocampus of Rats in Each Group

Compared with NC group, the expression of TNF-*α* mRNA, IL-1*β* mRNA, and IL-6 mRNA in the hippocampus of prop group rats was upregulated, and the content of TNF-*α*, IL-1*β*, and IL-6 in the hippocampus of prop group rats was upregulated (*P* < 0.05); compared with prop group, the expression of TNF-*α* mRNA, IL-1*β* mRNA, and IL-6 mRNA in hippocampus of minocycline group rats was downregulated, and the content of TNF-*α*, IL-1*β*, and IL-6 decreased (*P* < 0.05), as shown in Table 2.

### 3.5. Comparison of Cognitive Function of Rats in Each Group

Compared with NC group, prop group rats prolonged their escape incubation period on the 4^th^, 5^th^, and 6^th^ days (*P* < 0.05) and shortened their exploration time (*P* < 0.05). Compared with prop group, minocycline group shortened the escape incubation period and prolonged the exploration time on the 4th and 6th days (*P* < 0.05), as shown in Table 3.

## 4. Discussion

Hippocampus, as an important part of the central nervous system that is most closely related to cognitive functions such as learning and memory, is often damaged by external factors, resulting in cognitive dysfunction. Some scholars have found that propofol can block people's working memory and cause amnesia [19]. Animal models have also observed similar nerve damage effects of propofol, such as its effects on neuronal structure and cognitive function in rats, which are manifested as promoting neuronal degeneration and leading to cognitive dysfunction. In clinical work, propofol has been widely used in various outpatient diagnosis and treatment operations (such as painless gastrointestinal endoscopy) and anesthesia for daytime operations, with the proportion of elderly patients increasing year by year. Due to the short operation time, the patient can complete the operation with a single injection of propofol, so the patient will be discharged after the vital signs recover. However, the potential influence of propofol on the patient's cognitive function after the operation is often ignored, which lays hidden dangers for the patient's future rehabilitation. Rohan et al. [20] found that the incidence rate of POCD on the first day after cystoscopy or hysteroscopy under the anesthesia of a single anesthetic drug propofol or sevoflurane was 47%, which was higher than the incidence rate of POCD (26%) 7 days after major surgery reported in the past. Therefore, even if daytime surgery is performed under single drug anesthesia, the occurrence of POCD in elderly patients still deserves our high attention.

The article "Effects of Minocycline on Cognitive Impairment, Hippocampal Inflammatory Response, and Hippocampal Alzheimer's Related Proteins in Aged Rats after Propofol Anesthesia" was retracted in 2023. Reasons: suspected computer-generated content; unreliable results or conclusions; concerns about the data; concerns about the results or conclusions.

Some studies have shown that the upregulation of the expression of proinflammatory factors TNF-*α*, IL-1*β*, and IL-6 induced by narcotic drugs shows dynamic changes, but the expression of TNF, IL-1, and IL-6 is close to the peak value 6-24 h after anesthesia [21, 22]. Therefore, in this study, the mRNA expression level and protein content of proinflammatory factors 24 hours after anesthesia were measured. Although the excessive increase of proinflammatory factors lasts for a short period of time after anesthesia, some studies believe that the increase of proinflammatory factors caused by narcotic drugs can cause medium and long-term cognitive impairment. Therefore, this study chose to start cognitive function measurement on the 2nd day after anesthesia. In order to investigate whether minocycline regulates propofol-induced inflammatory response through GSK-3*β*/NF-*κ*B signaling pathway, Tau, and Amlyoid-beta, the expression levels of GSK-3*β*, acetyl-NF-*κ*B (Lys310), Tau, and Amlyoid-beta in hippocampus were further detected in this study.

The results of this study showed that the expressions of GSK-3*β*, acetyl-NF-*κ*B (Lys310), Tau, and Amlyoid-beta proteins in hippocampus of aged rats were upregulated after propofol treatment. The levels and contents of TNF-*α*, IL-1*β*, and IL-6mRNA were significantly increased. However, after preadministration of minocycline, it can inhibit propofol-induced upregulation of GSK-3*β*, acetyl-NF-*κ*B (Lys310), Tau, and Amlyoid-beta. The production of TNF-*α*, IL-1*β*, and IL-6 caused by propofol anesthesia is reduced. The behavioral performance of rats in MWM experiment was improved. It is suggested that preadministration of minocycline can improve the cognitive dysfunction induced by propofol anesthesia in aged rats [23]. The mechanism is that minocycline reverses the upregulation of GSK-3*β*, acetyl-NF-*κ*B (Lys310), Tau, and Amlyoid-beta expressions induced by propofol in hippocampus, thus affecting their transcription activity and reducing propofol-induced release of proinflammatory factors and inflammatory reaction.

The article "Effects of Minocycline on Cognitive Impairment, Hippocampal Inflammatory Response, and Hippocampal Alzheimer's Related Proteins in Aged Rats after Propofol Anesthesia" was retracted in 2023. Reasons: suspected computer-generated content; unreliable results or conclusions; concerns about the data; concerns about the results or conclusions.

## 5. Conclusion

In conclusion, preadministration of minocycline can improve cognitive impairment induced by propofol anesthesia in aged rats, and its mechanism of action may be related to minocycline inhibiting hippocampal inflammatory reaction and downregulating the expression of GSK-3*β*, acetyl-NF-*κ*B (Lys310), Tau, and Amlyoid-beta proteins in hippocampus.

## Figures and Tables

**Figure 1:** Comparison of GSK-3*β* and acetyl-NF-*κ*B (Lys310) protein expression in hippocampus of rats in each group (*n* = 5). Compared with NC group, a refers to *P* < 0.05, compared with prop group, b refers to *P* < 0.05. (a) Western blot was used to detect the expression of GSK-3*β* and acetyl-NF-*κ*B (Lys310) protein in hippocampus. (b) Semiquantitative analysis of GSK-3*β* and acetyl-NF-*κ*B (Lys310) protein expression in hippocampus.

**Figure 2:** Comparison of Tau and Amlyoid-beta protein expression in hippocampus of rats in each group (*n* = 5). Compared with NC group, a refers to *P* < 0.05, compared with prop group, b refers to *P* < 0.05. (a) Western blot was used to detect the expression of Tau and Amlyoid-beta protein in hippocampus. (b) Semiquantitative analysis of Tau and Amlyoid-beta protein expression in hippocampus.

**Table 1:** Comparison of arterial blood gas index and blood glucose of rats in each group (*n* = 5, $\bar{x}\pm s$).

Group	pH value	PaCO_2_ (mm Hg)	PaO_2_ (mm Hg)	Blood sugar (mmol/L)
NC group	7.36 ± 0.05	37.52 ± 3.19	112.51 ± 8.02	3.68 ± 0.52
Prop group	7.31 ± 0.04^∗^	38.47 ± 3.08^∗^	96.75 ± 4.63^∗^	4.17 ± 0.37^∗^
*P* value	1.034	1.244	0.995	1.231
Minocycline group	7.34 ± 0.05^#^	36.13 ± 2.75^#^	108.29 ± 8.34^#^	3.81 ± 0.35^#^
*P* value	1.225	1.432	0.998	1.242

Compared with NC group, ^∗^*P* > 0.05, compared with prop group, ^#^*P* > 0.05.

The article "Effects of Minocycline on Cognitive Impairment, Hippocampal Inflammatory Response, and Hippocampal Alzheimer's Related Proteins in Aged Rats after Propofol Anesthesia" was retracted in 2023. Reasons: suspected computer-generated content; unreliable results or conclusions; concerns about the data; concerns about the results or conclusions.

**Table 2:** Comparison of TNF-*α*, IL-1*β*, and IL-6 contents and mRNA expression in hippocampus of rats in each group (*n* = 5, $\bar{x}\pm s$).

Group	IL-1*β* mRNA	IL-6 mRNA	TNF-*α* mRNA	IL-1*β* (pg/g)	IL-6 (pg/g)	TNF-*α* (pg/g)
NC group	1.06 ± 0.07	1.03 ± 0.08	0.98 ± 0.04	27.34 ± 2.51	23.19 ± 3.05	31.63 ± 4.22
Prop group	3.35 ± 0.21^a^	2.97 ± 0.45^a^	4.42 ± 0.29^a^	55.72 ± 4.96^a^	44.18 ± 3.27^a^	78.51 ± 5.04^a^
*P* value	0.032	0.021	0.023	0.014	0.025	0.033
Minocycline group	1.24 ± 0.09	1.21 ± 0.07	1.13 ± 0.06	29.34 ± 3.18	24.06 ± 2.93	35.82 ± 4.27
*P* value	1.432	1.224	1.234	1.665	1.523	1.288

Compared with NC group, ^a^*P* < 0.05, compared with prop group, ^b^*P* < 0.05.

**Table 3:** Comparison of cognitive function of rats in each group (*n* = 10, $\bar{x}\pm s$).

Group	Escape incubation period					Exploration time
	At 2 d	At 3 d	At 4 d	At 5 d	At 6 d	
NC group	49.33 ± 4.26	41.47 ± 3.05	32.61 ± 2.32	21.97 ± 2.15	10.06 ± 2.83	41.75 ± 4.36
Prop group	54.52 ± 3.91^a^	48.35 ± 5.64^a^	45.83 ± 2.57^a^	37.16 ± 4.33^a^	30.18 ± 3.27^a^	22.16 ± 3.09^a^
*P* value	0.013	0.012	0.011	0.021	0.014	0.011
Minocycline group	54.06 ± 4.25^b^	43.27 ± 4.92^b^	30.11 ± 3.25^b^	20.24 ± 3.19^b^	12.37 ± 4.06^b^	34.95 ± 5.12^b^
*P* value	0.045	0.043	0.019	0.012	0.011	0.011

Compared with NC group, ^a^*P* < 0.05, compared with prop group, ^b^*P* < 0.05.

## Data Availability

The authors confirm that the data supporting the findings of this study are available within the article.
